The article "Computed Tomography Image Analysis of Body Fat Based on Multi-Image Information" was published in 2022. Journal: Biomed Res Int.

# Computed Tomography Image Analysis of Body Fat Based on Multi-Image Information

**DOI:** 10.1155/2022/8265211

**Published:** 2022-06-20

**Authors:** Wei Zang, Fengrui Zhu, Yang Yu

**Affiliations:** ^1^Department of 2nd Clinical College, China Medical University, Shenyang 110004, China; ^2^University of Surrey, 999020, UK; ^3^Department of Radiology, Shengjing Hospital of China Medical University, Shenyang 110004, China

## Abstract

Body fat assessment is required as part of an objective health assessment, both for nonobese and obese people. Image-based body fat assessment will enable faster diagnosis. Body fat analysis that accounts for age and sex will help in both diagnosis and correlating diseases and fat distribution. After evaluating computed tomography imaging algorithms to identify and segment human abdominal and subcutaneous fat, we present an improved region growing scale-invariant feature transform algorithm. It applies Naive Bayes image thresholding for key point selection and image matching. This method enables rapid and accurate comparison and matching of images from multiple databases and improves the efficiency of image processing.

## 1. Introduction

Obesity is a global health problem. Globally, 1.5 billion adults are overweight, and of these, 200 million men and 300 million women are obese. Child and adolescent obesity is increasing in both developed and developing countries, negatively impacting physical and mental health. According to the World Health Organization, global child obesity increased from 32 million in 1990 to 41 million in 2016. Obesity leads to metabolic syndrome and other complications, including type 2 diabetes mellitus, nonalcoholic fatty liver disease, hypertension, hyperlipidaemia, chronic kidney disease, cardiovascular disease, obstructive sleep apnoea, osteoarthritis, and malignant tumours (breast, colon, prostate, and others), thus increasing mortality [1].

Body fat imaging, which is crucial for diagnosis and research (Figure 1), has seen substantial advances in terms of field-of-vision and analysis. Reliable fat quantification is important in preventative healthcare and in diagnosing liver steatosis in nonalcoholic fatty liver disease, a risk factor for hepatocellular carcinoma development and progression [2]. Further, visceral obesity is an important predictor of metabolic syndrome, and measuring internal fat is important in understanding metabolic syndrome pathology. Nonetheless, there are as yet no unified diagnostic standards for fat detection.

Fat scanning methods include computed tomography (CT), magnetic resonance imaging (MRI), and ultrasound. Among these, only CT provides an accurate measurement of visceral fat area. Abdominal bioimpedance analysis (BIA), which is as accurate as abdominal CT, can safely and simply detect excessive visceral fat accumulation. Abdominal BIA is more effective than using waist circumference. Abdominal BIA has been used to study the connections between visceral fat area and metabolic syndrome risk factors. The characteristics of subjects with excessive visceral fat revealed via BIA, rather than via waist circumference, have been studied [3–5].

X-ray imaging, which led to unprecedented advances in diagnostic imaging, has a few disadvantages. In X-ray images, the pixel intensity is the sum of the attenuation of all the rays passing through the object, and three-dimensional results are projected on a two-dimensional plane. This inevitably duplicates information about the target's internal structure, preventing its clear display. CT imaging effectively overcomes this problem by scanning specific layers of the object and measuring the X-ray attenuation coefficient of the object at different angles. CT scanning provides multiangle data, enabling image reconstruction with reduced error. Computer-based reconstruction and algorithms enable the creation of multiple two-dimensional tomographic images.

Human abdominal fat comprises mainly visceral and subcutaneous fat. These two compartments with different molecular, biological, and anatomical compositions have a different meaning and importance. While subcutaneous fat shows a greater activity for long-term energy storage, visceral fat has a greater metabolic and hormonal activity through the release of adipokines [7]. Abdominal fat thickness is a risk indicator for conditions such as heart disease and diabetes. Although abdominal fat content, especially of intra-abdominal fat, is closely related to conditions such as type 2 diabetes, coronary heart disease, insulin resistance, and dyslipidaemia, the correlation between subcutaneous fat and these diseases is not significant [8, 9]. Measuring abdominal fat is more meaningful than measuring entire body fat. The body mass index, waist-to-hip ratio, waist circumference, and BIA are widely used to calculate and measure body fat. Waist circumference is widely accepted and used as an index of visceral fat.

Tetrapolar impedance measurement provides a simple and low-cost alternative method. Focused impedance, another method, provides local information. These two methods have been studied using an intuitive physical model and experimentally using a simulated abdominal subcutaneous fat layer. For accurate subcutaneous fat layer thickness measurement, tetrapolar and focused impedance require different electrode spacings. While small spacings between the current and potential electrodes hardly affect the impedance, larger distances reduce it substantially, until it becomes negligible. However, these methods require further analysis and experimental work [10].

For liver steatosis diagnosis and confirmation, complications are very rare. It is followed by histological classification based on the number of tissue cells with identifiable cytoplasm [11]. Although postbiopsy bleeding is a severe complication, there is a very low risk of massive haemorrhage if it is conducted carefully, and if patients are first screened properly. While such bleeding can occur unpredictably, it is related to age and malignancy [12]. Therefore, despite its advantages for determining visceral fat, the invasiveness and complications of biopsy provide motivation for developing noninvasive methods.

Ultrasound is fast and highly sensitive and has low negative effects on the human body. It is easily performed on comatose patients, which is an advantage with children, or with adults who cannot tolerate MRI, and has no sedative effect [13]. Abdominal obesity can be measured simply and economically via ultrasound and specifically via the newly developed quantitative ultrasound. In liver cirrhosis detection and measurement, quantitative ultrasound attenuation is determined based on the liver attenuation coefficient. It uses nonenhanced CT attenuation as the reference standard to enable noninvasive diagnosis and follow-up. However, ultrasound fat detection is not sufficiently intuitive and its results are difficult to store. The ultrasound device must be configured differently to detect visceral or subcutaneous fat. Because of these limitations associated with ultrasound imaging, CT and MRI are more widely accepted for visceral fat detection.

Compared to CT, MRI detects subcutaneous fat with similarly high consistency but with much greater error in visceral fat segmentation. Historically, nuclear magnetic resonance imaging has often been used to analyse visceral fat. For years, MRI has been considered the optimal noninvasive method for the assessment of fat accumulation [14]. However, it can disrupt cardiac metabolism, leading to complications; has low accuracy [15]; is slow; and is expensive, making it unpopular and uncommon. In human body, the classification of fat is not only subcutaneous and visceral but also white adipose tissue (WAT) and brown adipose tissue (BAT) according to its different functions. BAT is involved in energy dissipation and has been linked to weight loss, insulin sensitivity, and reduced risk of atherosclerotic disease [16]. Therefore, positron emission computed tomography (PET) has some advantages. For instance, 18F-FDG-PET/CT after cold exposure is the most commonly used and mature method for detecting and quantifying activated brown fat in the human body and evaluating its metabolic activity [17]. However, it is considered that PET has no significant effect on fat segmentation. The application of any radiotracer-based molecular imaging study in longitudinal studies with human subjects must take into account radiation dose [18]. So pet is not the main direction of fat segmentation.

CT, which has high repeatability, clinical safety, and convenience, produces high-resolution images and achieves accurate quantitative positioning [19]. Quantitative CT is therefore currently the technology-of-choice for body fat detection and analysis [20]. Nonetheless, it uses ionizing radiation, which limits repeated examination. Further, CT attenuation values based on voxels are confounded by the presence of substances such as glycogen, iron, copper, and iodine [21].

In this study, we analyse abdominal fat images (Figure 2), considering multiple factors, with the objective of elucidating human abdominal fat CT imaging. We examine various image segmentation methods and present an improved intelligent thresholding region growing segmentation method. We present a user-oriented graphical interface and examine image feature extraction and matching via scale-invariant feature transformation.

## 2. Materials and Methods

### 2.1. Image Segmentation

Image segmentation, central to image processing and developed over several decades, uses algorithms to decompose an image into several strongly correlated sets, segmenting the image into nonoverlapping areas. As with human visual cells, which separate objects from the background, digital image segmentation separates the objects as distinct areas of the image. Current techniques, using mathematical morphology, machine vision, intelligent algorithms, and other approaches, are based on segmentation thresholds, boundary extraction, and combined approaches.

Image segmentation, formally based on set analysis, strives to identify and extract the focal areas of an image. The entire image region is represented by the set *R*, which is divided into nonempty subsets *R*1, *R*2, *R*3, ⋯, *Rn*. Assuming that the two regions are critical, the union of *Ri* and *Rj* forms a connected region. *Ri* reflects regional connectivity, where *i* = 1, 2, ⋯, *N*. Neither the subregions nor regions intersect, and all pixels in the original image are within the union of all subregions. Connecting the pixels in each region in a defined way completes the segmentation process.

For all *i* and *j*, $i\neq \underset{¯}{j}$ and *Ri*∩*Rj* = ∅ holds; ∅ represents an empty set, and ∩ is the image set intersection. For *i* = 1, 2, ⋯, *N*, *P*(*Ri*) = true holds; *P* is a predefined attribute of *R*. Pixels in the same region should always have the same characteristics. Each subregion has unique characteristics: its elements must have the same grey level or similar characteristics. For *I* ≠ *j*, *P*(*Ri* ∪ *Rj*) = false holds; ∪ is the intersection. Pixels in different regions and subregions should have different characteristics, without common elements.

Most image segmentation algorithms are based on identifying discontinuity or similarity (consistency) in grey-scale images. Edge detection, which depends on abrupt changes in grey scale, is a typical example of discontinuity-based segmentation, while threshold segmentation, region growing, and other methods are based primarily on similarity. In edge-based segmentation, local grey-scale discontinuities between the background and boundary are integrated to detect the boundary. Alternatively, subregions can be separated based on background characteristics such as colour, texture, grey scale, or other unique properties. Segmentation should achieve smooth boundaries, and the pixels should be kept as smooth as possible within each region, without gaps. Irregular shapes can be smoothed using filter operators or algorithms that attempt to maintain boundary integrity. Adjacent regions should be effectively contrasted. Image segmentation methods differ in their principles and associated problems, and different methods are required for different fields.

The image sources are as follows: computed tomography (CT) images are stored in Digital Imaging and Communications in Medicine (DICOM) format. The normal images' sizes are 512 by 512. In this step, the DICOM images are converted to grey-scale portable network graphics (PNG) images. All images were standardized so that their pixel values lie in the range of [0,1]. The bed plate interferes with the separation process, so the subcutaneous fat will be automatically segmented after the histogram threshold is selected to remove the bed plate obstacle area.

### 2.2. Region Growing Segmentation

Region growing combines pixels or subregions into large regions, based on the nature of the problem, applying predefined growth criteria: it requires seed selection, a similarity criterion (growth rule), and a growth stop condition. The seed can be a single pixel or small area of several pixels. This algorithm forms sets of merged pixels with similar properties. For each region, a seed point is designated as the starting point; the surrounding pixels are compared with it, and similar pixels are merged until all similar pixels are merged. The similarity criterion can be based on grey scale, colour, gradient, and texture.

Further, connectivity must be considered in segmentation. Methods based only on texture or other similarity criteria can lead to false fusion or incorrect segmentation that has no research value.

#### 2.2.1. Seed-Point Selection

Seed pixels are selected to obtain seed points for regional growth. Change point selection can be automatic or based on semiautomatic (manual) human–computer interaction. Automatic selection can be targeted to field-specific image-analysis problems.

#### 2.2.2. Improved Region Growing Algorithm

Here, we present an improved region growing algorithm, which differs primarily from the other common region growing algorithms in its seed-point selection. Because fat and surrounding tissue do not differ sufficiently in contrast, it is difficult to select seed points using grey gradient maps. The improved algorithm first applies multidirectional automatic positioning of seed points among subcutaneous fat pixels, thus avoiding manual selection. Seed points are selected based on their grey features, on Euclidean distances between pixels, or via position analysis. In CT images, the subcutaneous fat boundary can usually be clearly identified, occurring between the dermis and the fascia and enclosed by the superficial fascia. Automatic seed-point selection enables the region growing algorithm to proceed effectively.

#### 2.2.3. Image Processing and Analysis

In CT images of body fat, the bed board appears in the lower part of the image, and its influence should be excluded to avoid meaningless segmentation. Because the location of the bed board is uncertain, there are more nonzero pixels in the subject area than in the obstacle area (Figure 3). By setting the threshold values for the nonzero pixels in the horizontal and vertical directions, based on analysis of the grey histogram in various directions, the uninteresting areas can be identified and excluded.

When selecting seed points, the improved region growing algorithm passes through eight directions of two main lines in the centre of the image and two diagonal sublines, and the rays from all directions converge at the centre of the image. The centre falls on the first nonzero pixel it meets; the growth thus proceeds several units in this direction into the subcutaneous region, thereby completing the first step of region growing.

Four grey-value ratios are then obtained, based on the grey values of the pixels in the four neighbourhoods around the seed point and on that of the seed point. At ratios greater than the predetermined similarity criterion, the points that meet the criterion can be included in the seed sequence; otherwise, growth is stopped. As the number of seed points increases, the grey value of the seed sequence approaches the average grey value of the subcutaneous tissue. As long as the grey-value ratio of the points in each new neighbourhood to that of the average for the image meets the predetermined conditions, the new neighbourhood is merged into the region. Thus, the average grey level of the sequence is updated and the region is grown. Once almost all of the subcutaneous fat pixels have been evaluated, the set of pixels represents the target fat area.

### 2.3. Intelligent Image Segmentation

Threshold analysis, which is computationally simple and generates intuitive results, can produce good results for images with large grey-value differences between the target and background. Various intelligent algorithms have been applied in machine vision to classify grey thresholds. Here, we used classical Bayesian classification to select the optimal grey-value threshold for fat images.

#### 2.3.1. Naive Bayes Algorithm

Image segmentation and classification are conventionally performed using the k-nearest neighbour's algorithm, neural networks, and decision trees. Bayesian classification applies Bayes' probability theorem (a class of intelligent algorithms) to categorise objects by their characteristics. Among such classification methods, Naive Bayes is the most efficient and effective, in some cases performing better than neural networks and decision trees.

The Naive Bayes algorithm, which is mathematically derived, is based on clear rules that are easy to understand. Further, it is easier to specify and debug than other methods. It is widely applicable and rapid to implement, accepts most types of data, and is computationally efficient. In Bayesian classification models, the potential default attribute is independent. While this constrains its use somewhat, it also reduces its complexity and resource requirements.

#### 2.3.2. Segmentation Analysis

Naive Bayes classification classifies items by placing them in the category with highest probability, under this condition. The initial threshold is the average of the minimum and maximum grey levels. The grey values and numbers of the pixels with grey values above or below the initial threshold are then obtained, for all images. The grey values and numbers of pixels on each side of the points between the threshold values are summed to obtain the total grey values above and below the initial threshold values and averages. An iterative threshold optimisation algorithm is then applied; after each iteration, the target threshold value is approached from the direction that increases the existing threshold probability value. The iteration continues until the difference between the front and back threshold values is close to 0, finally returning the optimal threshold value (Figure 4).

Although the optimised segmentation threshold is close to the ideal threshold, many connections between visceral and subcutaneous fat points are broken during the optimization process. Further, the segmentation is affected by the presence of many connections between the external boundary and the background.

### 2.4. Fat Image Analysis Based on Scale-Invariant Feature Transformation

#### 2.4.1. Scale Invariant Feature Transform (SIFT) Algorithm

The SIFT algorithm (patented by David G. Lowe), which assumes that two photos contain the same content, applies affine transformation based on the degree of illumination, image angle, and size. It aims to match two points in the two images.

The SIFT algorithm recognises objects by extracting key points, creating corresponding descriptors, and identifying corresponding feature points via matching, thereby connecting the corresponding points (Figure 5). SIFT features are not affected by ordinary affine transformation and differences in image brightness and are relatively unaffected by noise. SIFT is thus suitable for accurate and fast image matching. Even when there are several objects in the same area, it generates many SIFT feature vectors.

For images of body fat, SIFT can match CT images of the same person at specific points. The ability to match processed body fat CT images to their corresponding database images, via feature point matching, will substantially improve diagnostic efficiency. This method thus contributes to the database and represents an advancement in image processing.

#### 2.4.2. Scale-Space Construction

Before the SIFT algorithm is implemented, the scale space must be constructed (Figure 6); on the left-hand side of the figure is the Gaussian pyramid model, with several explanations. Gaussian convolution is one manifestation of scale space, and Gaussian blur is widely used to analyse scenes where it is necessary to reduce the size. Octaves represent groups of images of the same size. Images are processed by interval within each octave; scales within the scale space are interpreted as groups, and the image blur of each group gradually increases from bottom to top.

A Gaussian kernel, which is required to generate a multiscale space, simulates clarity for near objects and ambiguity for distant objects [22]. To calculate Gaussian kernels with different variances, the original image is convolved with Gaussian kernels of different sigma, to obtain all the first-group (bottom) layers. The Gaussian pyramid is thus obtained by convolving the original image sequentially, via Gaussian kernels of different scales. The second group of images is obtained by down sampling the first group via interval sampling, which maintains a continuous scale. A single pixel has little influence on the whole image.

The normalised LOG operator is scale-invariant [23]. The LOG operator is related to differences in Gaussian kernel function, giving rise to the Gaussian difference operator. The Gaussian difference pyramid is obtained by subtracting one layer from its adjacent layer in the same group (right side, Figure 7). Gaussian difference calculation requires Gaussian smoothing of adjacent scales.

#### 2.4.3. Accurate Key Point Positioning

After image thresholding, the extreme values must be detected. Local extreme value points in the Gaussian difference space constitute the key points. Key points are generally relatively stable, providing much information, and are used in image matching. They are usually retained even when external conditions change, appearing as bright points in dark areas or dark points in bright areas.

In Figure 8, the X point of the middle layer is compared with eight adjacent points in the same scale space and 18 vertically adjacent points, totalling 26 points. Every pixel is compared in the same way. After finding the extreme value points, they must be accurately located. The extreme value points and scale space are discrete at this stage. Applying ternary second-order Taylor expansion to the detected extreme value points and adjusting their positions improve their subpixel location accuracy. The number of iterations is limited. Points with low contrast (values <T/N) are removed; T is generally 0.04. In addition, to ensure feature point stability, the Gaussian difference edge response must be eliminated.

#### 2.4.4. Constructing Key Point Direction

The selected key points, which are relatively accurate, are characterised by their *X*, *Y*, and *σ* (scale) parameters. We first find the image closest to the *σ* value of the key point scale in the Gaussian pyramid and draw a circle with the point as the centre and radius 1.5 times the Gaussian image scale (Figure 9). Accounting for the gradient direction and gradient amplitude of the pixels in the circle, the whole angle is divided into eight directions. There are improved methods that select one direction every 10° in a 360° histogram, thus generating more than eight directions. In that case, 1.5*σ* Gaussian filtering is then applied.

To finalise the key point detection, the most frequent direction from the previous iteration is selected as the primary direction (Figure 10). Feature points have at most one auxiliary direction. A feature point with two feature directions is regarded as two feature points (one main and one auxiliary feature point), with the same position and scale, but different directions.

#### 2.4.5. Key Point Descriptors and Matching

Key points have four parameters, namely, *X*, *Y*, *σ* (scales), and main direction (Figure 11). Pairs of images are matched using a descriptor, which describes the key point using a set of vectors. The descriptor contains both the key point and surrounding pixel points, which may contribute to target matching. The unique vector is generated by dividing the region into blocks and calculating the gradient histogram for each block. Typically, 128-dimensional vector representation is the most advantageous.

Once the descriptor area is determined, it is converted to the main direction. Using the KD tree algorithm or the more efficient K nearest-neighbour algorithm, the descriptors of all key points in the two images are extracted, and the two descriptors with the shortest distance are selected. These two descriptors may be for the same key point. The gradients in eight directions are then counted in each subregion.

## 3. Results and Discussion

### 3.1. Matching of Parts with the Whole

With the exception of some fuzzy edge points, the key points and image registration were accurate (Figure 12).

There was a high degree of registration between the local image in the edge area and the whole image; further, the part cut from the right part area was consistent with the part of the original image matching the feature points (Figure 13).

### 3.2. Matching within and between Groups

Images in the same group came from one individual. Therefore, we conducted matching within groups to screen feature images for this individual in the database. There were 436 matched features, showing high matching accuracy (Figure 14).

We conducted feature matching of abdominal fat images from different groups (individuals). There were 21 matched features between these different groups (Figure 15), substantially less than the 436 matched features within the same group.

### 3.3. Data Analysis

Based on SIFT image registration, we conducted partial and overall analyses and intra- and intergroup analyses. The former analyses the key points, matches, and time parameters of the registration between the parts and whole, by list. The latter provides inter- and intragroup comparisons of the three groups. The mean key point value was 498.5, the average number of matches was 30, and the average matching time was 0.235 s (Table 1). This algorithm performs fast, identifying ca. 500 key points in each group and ca. 30 matches. To ensure proper representation, we selected six groups of CT images (that is, from six individuals) and registered and compared the whole and parts.

The left of the histogram (Figure 16) shows the contrast registration number of the same group, and the right shows the configuration number between different groups. We set up three control groups. From the control group histograms, it is clear that image registration was high within groups but low between groups.

The main file generated by the algorithm comprised of the input image Gaussian scale and difference spaces, local extreme value selection, and key point descriptor calculations based on the image gradient.

## 4. Conclusions

This study presented an improved region growing scale-invariant feature transformation algorithm for human body fat image segmentation and image registration. It used a Naive Bayes classification algorithm for intelligent threshold segmentation. It applied multidirectional convergence and automatic positioning of seed points, advancing semiautomatic manual seed-point positioning. As the seed points expanded, the region grew according to a ratio-similarity growth rule, until the subcutaneous fat region was completely segmented. Given the complexity of visceral tissues, and the abundance of connections between internal fat pixels, we did not examine visceral fat imaging in more detail.

This improved algorithm effectively matched the images within groups (individuals) based on feature similarity, in both the part-to-whole and intragroup registration tests. It has broad operational significance and performs better than other segmentation algorithms. This improved registration of human body fat CT images therefore advances image analysis and makes this algorithm more applicable for research. It provides a conceptual basis for future imaging research.

In the submission, we did not give the corresponding design and application, but in other articles we designed a “one-click segmentation” operation for the quick segmentation of fat images for the convenience of the users. The segmented image is obtained directly after the user interacts with the user interface (UI) component, and there are other useful operations for the user to handle the image.

The “one-click segmentation” operation includes functions such as opening and saving files, setting fonts, printing settings, specifying prompt messages, and entering commands. After the user selects the image in the computer library, the program will read in the image and the user can perform the crop step. The program will eventually show the results of processing the original image for this project and other images in interest. The user can directly see the processing results of various operators through this detection function, and it is easy for the user to learn and discuss. After use, the user can also save and print the results, which can make the user feel the shortcut of the program, whether it is teaching or research.

## Figures and Tables

**Figure 1:** Relationships between obesity, visceral fat, cardiovascular disease, liver steatosis, metabolic syndrome, and nonalcoholic fatty liver disease [6].

**Figure 2:** Manual segmentation of human fat CT images.

**Figure 3:** Segmentation based on the original and improved region growing algorithms.

**Figure 4:** Comparison of segmentation result using the Bayesian algorithm.

**Figure 5:** Implementation of the scale invariant feature transform (SIFT) algorithm.

**Figure 6:** Gaussian difference pyramid model [23].

**Figure 7:** Construction of the Gaussian difference pyramid [23].

**Figure 8:** Extreme value point selection [22].

**Figure 9:** Image gradient of the area around the key points [22].

**Figure 10:** Histogram of key point direction.

**Figure 11:** Axis direction transformation [22].

**Figure 12:** Feature matching between the central and whole region of the human abdominal fat image.

**Figure 13:** Image registration of the edge area and the whole area of CT images of human abdominal fat.

**Figure 14:** Image matching within the same group.

**Figure 15:** Image matching between human body fat images from different individuals.

**Figure 16:** Comparison of the SIFT registration number between groups of CT images of human abdominal fat.

**Table 1:** SIFT registration of the parts and whole of CT images of human abdominal fat from six groups (individuals).

Group	Key points	Matches	Time
1	324	20	0.124
2	428	27	0.232
3	683	33	0.353
4	564	26	0.257
5	477	36	0.296
6	515	38	0.153
Mean	498.5	30	0.235

## Data Availability

All data included in this study are available upon request by contact with the corresponding author.
